# Deep Learning-Based Medical Information System in First Aid of Surgical Trauma

**DOI:** 10.1155/2022/8789920

**Published:** 2022-04-16

**Authors:** Yong Liang, Yugeng Liu, Bo Liu, Aimin Xu, Junyu Wang

**Affiliations:** ^1^Department of Emergency, Beijing Chao-Yang Hospital, Capital Medical University, Beijing 100043, China; ^2^Emergency Medicine Clinical Research Center, Beijing Chao-Yang Hospital, Capital Medical University, Beijing Key Laboratory of Cardiopulmonary Cerebral Resuscitation, Beijing 100043, China

## Abstract

The aim of this study was to explore the application of process reengineering integration in trauma first aid based on deep learning and medical information system. According to the principles and methods of process reengineering, based on the analysis of the problems and causes of the original trauma first aid process, a new set of trauma first aid integration process is established. The Deep Belief Network (DBN) in deep learning is used to optimize the travel path of emergency vehicles, and the accuracy of travel path prediction of emergency vehicles under different environmental conditions is analyzed. DBN is applied to the surgical clinic of the hospital to verify the applicability of this method. The results showed that in the analysis of sample abscission, the abscission rates of the two groups were 2.23% and 0.78%, respectively. In the analysis of the trauma severity (TI) score between the two groups, more than 60% of the patients were slightly injured, and there was no significant difference (*P* > 0.05). In the comparative analysis of treatment effect and family satisfaction between the two groups, the proportion of rehabilitation patients in the experimental group (55.91%) was significantly better than that in the control group, and the satisfaction of the experimental group (7.93 ± 0.59) was significantly higher than that of the control group (5.87 ± 0.43) (*P* < 0.05). Therefore, integrating Wireless Sensor Network (WSN) measurement and process reengineering under the medical information system provides feasible suggestions and scientific methods for the standardized trauma first aid.

## 1. Introduction

With the development of the national economy, the application of modern tools and machinery has expanded, and with the increase in traffic accidents, the trauma problem has become an important factor that jeopardizes the health of the people, posing great challenges to the medical community. Trauma first aid plays a very important role in the whole emergency medicine. The success rate of trauma first aid not only reflects the hospital's own technical level but also is an important indicator to measure the medical level of the whole country [1–3].

With the deepening of the medical system reform, competition between hospitals has become increasingly fierce. The emergency department is a window for the hospital to face the society. Its workflow and quality directly affect the image and comprehensive strength of the hospital [4, 5]. As the most direct digital medical equipment to high-level information and knowledge sharing, the medical information system has directly or indirectly improved the ability of medical diagnosis and treatment. Exploring the medical service model suitable for the actual situation of the hospital and formulating a feasible integrated trauma first aid process capable of continuous quality improvement are an urgent need to adapt to the development of the hospital and face the continuous reform and deepening of the medical system [6–8]. In the implementation of first aid, shortening the transportation time of patients by ambulances can also effectively improve the treatment effect of patients. Many researchers have studied it. Wang et al. evaluated a patient-centered electronic comprehensive status display, which was aimed at supporting clinicians in the emergency departments (EDs) of the hospital to communicate and realize the health status and progress of patients through their ED care plan [9]. Duguid et al. investigated the potential of ward electronic drug distribution cabinet to provide patient-level data and be alert that antibiotics were not used in hospitals. It was found that the electronic drug distribution cabinet report had proven to be useful to promote good antibacterial management in general hospitals [10]. The application of an electronic medical system in trauma first aid has shown its advantages. Meanwhile, the application of deep learning in path planning has been proven to have good performance.

Based on the support of medical information technology, the problems existing in the original emergency treatment process are analyzed and a new comprehensive emergency treatment process is established. Moreover, it is applied to clinical surgery in hospital to verify the applicability of this method and prove that this emergency treatment process can shorten the treatment time of trauma patients, enhance the treatment effect, and improve the satisfaction of patients' families.

## 2. Wireless Sensor Network Measurement and Medical Information System Assisted Process Reorganization to Build an Integrated Trauma Emergency Process

### 2.1. Research Methods

After analysis, this study comprehensively applies systematic reintegration and partial process reengineering methods, examines the traditional surgical trauma first aid process [11], and conducts semistructured qualitative interviews with relevant staff in the emergency department to discover the unreasonable links in the traditional surgical trauma first aid process and affect the emergency department. The key quality control points of quality classify the causes and make full use of the latest research results of information technology and literature, improve and reorganize the old process according to the theory and methods of process reorganization, and form an integrated trauma emergency process [12]. We, after consultation with relevant experts, revised and improved the first draft, formed the final draft of the integrated trauma first aid process and through the experimental research studied the application effect of the new process, and constructed the integrated trauma first aid process circuit diagram as shown in Figure 1.

### 2.2. Traditional Surgical Trauma First Aid Process

The description of the traditional trauma first aid process is shown in Figure 2.

As shown in Figure 2, the specific process flow is described as follows. (1) After dispatching the police to 120, the doctor and nurse from the clinic will get out of the car within two minutes. (2) After the medical staff arrives at the scene, judge whether the surrounding environment is safe and judge the patient's condition and state of consciousness. (3) For patients who need CPR or defibrillation, in addition to general treatment such as pressure bandaging and establishment of venous access, CPR and defibrillation should be performed on site and patients should be taken back to the hospital at the fastest speed. (4) For general patients, general treatment is used, such as establishing venous access, compression dressing, pain relief, etc., and then returning to the hospital for treatment. (5) After the shock patient enters the hospital, the medical staff urgently prepares the bed unit, prepares the tracheal intubation, suction device, and other rescue items, opens the green channel, rescues first, and then charges. After the rescue, transfer to the emergency operating room or intensive care unit. (6) After the general patient enters the hospital, the triage nurse performs the triage, the emergency doctor collects the medical history and conducts the physical examination, and the family members go through the registration procedure. The emergency doctors prescribe the laboratory according to the patient's condition and the radiology examination, and the family members pay the relevant fees after the payment. The overall flow is “division-registration-visit-payment-payment-inspection-diagnosis~payment-treatment.” (7) Ask the relevant professional doctor for an emergency consultation and the necessary treatment. The necessary treatment is performed in the emergency department, and the patient is diverted to the relevant surgical ward, intensive care unit, emergency operating room, interventional operating room, etc. according to the opinion of the specialist and emergency doctor [13].

### 2.3. Problems with Traditional First Aid Procedures

(1) Some outpatient medical staff have insufficient experience in dealing with acute trauma patients. (2) Prehospital emergency equipment is not perfect. (3) Critically ill patients wait for a longer consultation time. (4) There is insufficient hospital preparation for patients requiring shock recovery. (5) There is no tacit understanding between the medical staff during the recovery. (6) There is no priority for the payment of the first-level patients. (7) Some of the emergency indicators are slow to test. (8) There is no uniform standard for the treatment process in the hospital. (9) The patient waited longer for admission. (10) There are many patients in the hospital, and the monitor often becomes insufficient.

## 3. Design New Process

### 3.1. Process Procedure

Based on the concept of process reengineering, the research team adopts methods such as optimizing core links, vertical linkage in the front yard, and multisector horizontal cooperation. Based on the expert opinions, combined with the current situation of the department, the integrated trauma first aid process (first draft) is shown in Figure 3.

(1) After dispatching the police to 120, the doctors and nurses who have been trained in trauma treatment will get out of the car within two minutes. (2) After the medical staff arrives at the scene, judge whether the surrounding environment is safe and judge the patient's condition and state of consciousness. (3) For patients who need CPR or defibrillation, in addition to general treatment such as pressure bandaging and establishment of venous access, CPR and defibrillation should be performed on site and patients should be taken back to the hospital at the fastest speed. Improve prehospital first aid equipment, increase transshipment stair stretchers, reduce transit time, and prevent secondary injuries. The ambulance is equipped with a ventilator to improve the success rate of shock patients. (4) For patients with shock, contact the hospital outside the hospital and contact the relevant department physician in advance to wait for the patient to consult [14]. Contact the emergency department outside the hospital, prepare for recovery, and open a green channel. The rescue room has a fixed recovery area, and the positioning and rescue are carried out. The positions of the personnel are fixed, and each performs its duties to improve the rescue efficiency. For general patients, general treatment is used, such as establishing venous access, compression dressing, pain relief, etc., and then returning to the hospital for treatment. (6) After the general patient enters the hospital, the triage nurse performs the triage, the emergency doctor collects the medical history and conducts the physical examination, and the family members go through the registration procedure. The emergency doctors will open the laboratory according to the patient's condition and perform the standardized trauma patient treatment process, and the radiology examination will be carried out after the family members pay the fee. When the family members pay the fee, the toll booth sets a green channel for the first-level patient payment and preferentially pays for the first-level patient. The consultation process is integrated into “division-visiting-registered-prepayment-inspection-diagnosis-treatment-integrated payment” to save the patient's family from unnecessary intermediate links and waiting for queuing time. The emergency department adds additional bedside rapid testing equipment, such as blood gas analyzers, to speed up the inspection. (7) Ask the relevant professional doctor for an emergency consultation and the necessary treatment. The necessary treatment is performed in the emergency department, and the patient is diverted to the relevant surgical ward, intensive care unit, emergency operating room, interventional operating room, etc. according to the opinion of the specialist and emergency doctor. Improve the equipment of debridement and suture room, equipped with a shadowless lamp, operating bed, anaesthesia hanging tower, etc., so that some patients with mild trauma can be cured in the emergency department. Increase the number of juries and shorten the waiting time for patients [15]. (8) The WSN-based vital sign monitor is used to measure the vital sign data (the patient's temperature and heart rate) and alarm the data beyond the normal range. The monitor consists of a sensing node and a basic node. The sensing node includes a wireless transceiver module, a body temperature sensor, and a heart rate sensor. The sensor node is worn on the patient, and its microcontroller measures and receives the vital sign signals such as the heart rate and body temperature of the patient. Then, the signals are transmitted to the wireless network for data processing and storage. The processed data are displayed with a graphical interface, which is convenient for medical personnel to perform vital sign signal analysis.

### 3.2. First Aid Route Optimization Based on Deep Learning

In this study, DBN was adopted to find the optimal route of emergency ambulances in the process of first aid. The DBN is mainly composed of multiple restricted Boltzmann machines, and the basic structures of the restricted Boltzmann machine and the DBN model are shown in Figure 4.

When treating patients with first aid, the proper planning of the 120 ambulance first aid route can markedly save the overall time of first aid. In the planning of the emergency route, the key point is the effective prediction of the current road traffic conditions of the road section that the emergency passes through, and then, the emergency route is selected based on the predicted road conditions. The basic process of using deep learning for route planning of emergency ambulances is shown in Figure 5.

The prediction of traffic network conditions needs to consider factors such as weather, road construction conditions, holidays, and rush hours. The new version of the meteorological disaster warning signal has revised the original 5 grades into 4 grades, which are blue (normal), yellow (heavier), orange (serious), and red (particularly serious). Therefore, the image value of weather was divided into 4 regions in this study. Assume that the cost value of traffic during the working day and under normal weather conditions was defined as the standard value *T*_0_ and the cost of warning weather was *T*_*w*_, and the calculation of the weather influence value *T*_*i*_ is shown in

(1) $$\begin{array}{c} T_{i}=\frac{T_{w}}{T_{0}}\;\left(w=1,2,3,4\right). \end{array}$$

The national traffic regulations stipulate that the speed limit for roads without a centerline in the city is 30 km/h, and it is 40 km/h for highways. In order to facilitate the subsequent calculation, the road was divided into two categories in this study, namely, the maximum speed of 40 km/h and the minimum speed of 0 km/h, and the state value of the road was set as RbR.

Since the data in this study were divided by hour, the impact of peak commute and weekends could be ignored. The influence value *V*_*i*_ of holidays was the ratio of *T*_0_ to the generation value *V*_*w*_ under the influence of weather, which could be calculated in

(2) $$\begin{array}{c} V_{i}=\frac{V_{w}}{T_{0}}\;\left(w=1,2,3,4\right). \end{array}$$

Then, a deep learning model based on the self-encoding network was applied to calculate the weight of the hidden layer in the network. The solution of the weight value in the model adopted the gradient descent method, and the solution process was as follows.

(3) $$\begin{array}{c} \left\{\begin{array}{c} z=\omega^{T}v+b,\\ f\left(z\right)=\frac{1}{1+\exp\left(-z\right)}. \end{array}\right. \end{array}$$

In equation (3), *ω* stood for the weight value of the hidden layer, *v* represented the input feature vector, and *b* meant the bias.

The softmax prediction model was employed to classify the results, and the cost function is expressed in

(4) $$\begin{array}{c} v\left(\theta \right)=-\frac{1}{m}\left[\overset{m}{\underset{i=1}{\sum }}\overset{k}{\underset{v=1}{\sum }}1\left\{y_{i}=v\right\}\log\frac{e^{\theta_{v}^{T_{x}^{\left(i\right)}}}}{\sum_{v=1}^{k}e^{\theta_{v}^{T_{x}^{\left(i\right)}}}}\right]. \end{array}$$

*m* refers to the data sample size and *k* indicates the number of sample categories. The optimal route selection for first aid needs to follow the following principles. The first one is the shortest path; that is, the total length of the road section that the 120 ambulance passes through is the shortest. The second one is the shortest time; that is, the 120 ambulance reaches the location of the patient and sends the patient to the designated hospital within the shortest time. The third one was that the path is feasible; that is, the selected path does not have problems such as road closure and serious congestion. Based on this, the mathematical expression of route weight proposed in this study was as follows.

(5) $$\begin{array}{c} w=L\times T_{i}\times V_{i}\times v\left(\theta \right)\alpha . \end{array}$$

In equation (5), *L* and *α* stood for the total length of the road section and a fixed coefficient, respectively.

### 3.3. Description of Key Links in the Reorganization Process

1. Establish an independent emergency medical team and improve its overall quality

First of all, improve the comprehensive consultation ability of the team of doctors. Due to the nature of emergency medical services and the specificity of emergency departments and emergency diseases, first aid tasks require high, full, and fast access to doctors, which requires a high degree of responsibility. It is generally believed that for an emergency physician, sense of responsibility is more important than medical technology. Second, comprehensive medical knowledge and superb medical technology are required to be familiar with the diagnosis and treatment of various emergencies, to be agile and correct in operation, to be good at grasping major contradictions, and to take effective measures to save the lives of patients. Through prejob training and practice, it is required to master various first aid technologies, such as basic life support technology (BLS), advanced life support technology (ACLS), and primary trauma treatment technology (PTC). To enter the emergency team, it is necessary to go through the rotation of each area in the emergency department, including training in areas such as prehospital emergency, emergency general examination area, emergency observation area, and emergency rescue area. It also requires going through strict assessment, including the treatment of various acute diseases.

In the training of emergency nurses, the overall quality of the trauma emergency nurse team is improved from the whole process of emergency treatment, including outpatient nurses, triage nurses, rescue nurses, and emergency surgery nurses, especially for young nurses and new nurses. Prejob training and practical guidance enable them to quickly detect the condition and to have timely observation, accurate response, and proper coordination with doctors to improve emergency first aid efficiency and shorten treatment time.

(2) Establish a standardized trauma emergency procedure

The first is the prehospital visit. When receiving a serious traumatic outpatient task such as multiple injuries, immediately dispatch a senior medical staff member in the duty team to visit the doctor. Immediately after the emergency personnel arrived at the accident site, the injury was quickly assessed. The airway, respiratory, circulatory, and neurological dysfunction and systemic exposure were quickly assessed according to PTC requirements. After the haemostasis, dressing, and fixation, the prehospital trauma index score was applied. The patient is scored and informed of the pre-hospital treatment, and the specialists are contacted to prepare as soon as possible.

Followed by on-site processing, the on-site processing process is standardized, mainly using PTC sequential evaluation and TI scores. TI score of 2-9 indicates minor injury. Emergency treatment or observation, debridement and suture, and anti-infection treatment were carried out through consultation and shunt. TI score of 10-17 indicates moderate injury, i.e., stable vital signs and suspected potential injury. After thorough examination, such as chest piercing, abdominal wear, and imaging examination, go through the hospitalization procedures and send them to the corresponding ward for elective surgery. TI score of 17-20 indicates serious injury. With multiple injuries, the mortality is high. The examination should be carried out as soon as possible, antishock and preoperative preparation should be carried out simultaneously, and the patients should be accepted into the intensive care unit or directly into the operating room. TI score > 20 indicates fatal trauma, including massive hemorrhage, asphyxia, and pneumothorax. Emergency surgery or injury control surgery should be performed immediately. According to the patient's condition, the patient is placed in the rescue area, observation area, and general surgical area [16].

(3) Synchronous transmission of patient information

Introduce an emergency information system to integrate emergency triage, rescue, observation, treatment, and charge, share patient information, reduce manual error rate, realize synchronous transmission of HIS, LIS, and PACS programs, and enable emergency doctors to obtain inspection results in the shortest time. Speed up the diagnosis and treatment, and avoid patients and their families from going to and from the emergency areas and examination rooms, avoiding multiple queues and repeated payment. Through the remote audio and video system, the prehospital physician informs the patient in advance, informs the hospital to receive the consultation, and reduces the phenomenon of pushing the department, and the relevant specialists prepare early and enter the emergency department for waiting.

## 4. Evaluation of Recombination Procedures in Surgical Trauma First Aid

### 4.1. Object Selection

From January to December 2018, the patient was taken back by the 120 ambulance of hospital. The patient who was admitted to the hospital for diagnosis by trauma was the experimental group. The trauma patients who were treated in hospital were selected as the control group. Relevant information of the medical records of the control group was collected by retrospective investigation. The study had been approved by the ethics committee of the hospital, and the subjects knew the content of the study and signed the informed consent.

Inclusion criteria were as follows: (1) trauma occurring until admission time < 24 h, admitted to hospital for emergency trauma; (2) age 18 years old: (3) causes of traffic injuries, fall injuries, crush injuries, sharp injuries, and trauma; and (4) prehospital electronic medical records and in-hospital emergency records being clear. Exclusion criteria were as follows: (1) patients who were transferred halfway and (2) patients who gave up treatment by themselves and their families. The estimation method is based on the sample size in an experimental study:

(6) $$\begin{array}{c} {\text{n}}_{1}=n_{2}=2\times {\left\{\frac{\left(u_{\alpha }+u_{\beta }\right)\sigma }{\delta }\right\}}^{2}. \end{array}$$

And refer to the relevant study in the emergency trauma patients' access diagnosis and treatment time *δ* value and standard deviation *σ* calculated about 110 cases per group, taking into account 15% of the rate of loss to follow-up (n_1_ = *n*_2_ = 125 cases).

### 4.2. Measurement Tools

1. Patient general information questionnaire. The researcher designed the study according to the purpose and content of the study, including the sex, age, and cause of the trauma, the time from trauma to admission, and the time from admission to diversion
2. Time points for various rescues. The time points of the visits and rescues included in the study were time of departure, time of arrival, time of on-site treatment, average transit time, average on-the-go standby time, and average mission time
3. Patient family satisfaction score. The patient's family satisfaction scale is divided into three aspects: medical work service attitude, first aid project satisfaction, and treatment effect satisfaction. The scores correspond to very satisfied (3 points), basically satisfied (2 points), neutral (1 point), and dissatisfied (0 points)

### 4.3. First Aid Method for Injured Patients

In the control group, the first aid patients were treated with traditional treatment mode, as shown in Figure 3. The patient's trauma first aid method in the experimental group is shown in the gravy background standard part of the process. The detailed description is given in the second part.

### 4.4. Analysis Method of Data

The data processing and analysis were carried out by using SPSS22.0 statistical software. The statistical methods used were descriptive statistics, chi-square test, *τ*-test, *z*-test, etc. The test level was taken as two sides *α* = 0.05. *P* < 0.05 showed that the difference was statistically significant.

### 4.5. Quality Control

This study focuses on quality control in several key aspects of research implementation, such as consulting first aid clinical and nursing experts when constructing an integrated trauma first aid process to ensure the reliability and scientific nature of the process: in the data collection phase, especially it is the investigation of the patient's family satisfaction questionnaire. The unified training investigator completes the method of on-site recovery. In the processing stage of statistical data, further consult the relevant epidemiologists and statistics experts to ensure the correctness and professionalism of the analyzed data [17, 18].

## 5. Results

### 5.1. Sample Shedding

After screening, 134 cases were finally included in the intervention group and 3 cases fell off. The reason of losing follow-up was that 2 cases gave up treatment and 1 case lost to follow-up due to contact change; 128 cases in the control group were included, and 1 case fell off. The reason was that the data analysis did not conform to the principle of logical inspection. The abscission rates between groups were 2.23% and 0.78%, respectively.

### 5.2. Comparison of Data between the Two Groups of Patients

The experimental group, with a total of 127 cases, has the average age of 45.67 ± 16.19 years. There were 131 patients in the control group with an average age of 47.62 ± 19.51 years. There was no significant difference in age between the two groups before and after the recombination (*t* = 0.179, *P* > 0.05). There were no significant difference in gender between the two groups (0.274, *P* = 0.605 > 0.05) and no statistical significance in the cause of injury (0.613, *P* = 0.716 > 0.05). The baseline data of the two groups of patients were balanced and comparable, as shown in Table 1.

### 5.3. Comparison of Wound Index Scores between the Two Groups

Comparison of TI scores between the two groups is shown in Table 2. In the control group, 79 patients scored 2-9, 32 patients scored 10-17, 12 patients scored 17-20, and 8 patients scored 20 or above; in the experimental group, 77 patients scored 2-9, 33 patients scored 10-17, 12 patients scored 17-20, and 5 patients scored 20 or above. There was no significant difference in the preschool TI score between the two groups in the rank sum test (*χ*^2^ = 0.469, *P* = 0.931 > 0.05).

### 5.4. Verification of Emergency Route Planning Based on Deep Learning

The specific process of using deep learning technology to realize the route planning of emergency ambulances in the process of first aid was as follows. First, the input data were screened out and grouped according to the time period, which were eventually classified into normal weather+working days (standard), warning weather+working days, and normal weather+holidays. Second, the standard data were applied to train the deep learning model, and the output characteristics of the model were determined, so as to calculate the cost value *T*_0_ of the standard road section. Third, the classified data were trained and each predicted cost value was solved, such as weather influence value *W*_*i*_ and holiday influence value *V*_*i*_. Fourth, the standard time-sharing data was adopted to learn the deep learning model, and solve the cost value *T*_0_ and coefficient *α* of different road sections. Fifth, the road section cost value *T*_0_ and influence value at the corresponding time were selected according to the distribution information, which were brought into equation (5) to construct a weighted traffic network. Sixth, the emergency search algorithm was used to solve the optimal route in the weighted traffic network. Seventh, the optimal route for first aid was eventually output.

The traffic data information was collected for screening and classification, and the traffic data were randomly divided into 3 groups, namely, comparison group 1, comparison group 2, and standard group. Each group of data contained 10,000 samples. After obtaining the characteristic information of the data, there was full-time prediction of the model, thus calculating the impact factors of weather, working days, and holidays and testing the model. The prediction accuracy of this model is shown in Figure 6. It was found that the average prediction accuracy rates of *T*_0_ (Figure 6(a)), *W*_*i*_ (Figure 6(b)), and *V*_*i*_ (Figure 6(c)) were 80.2%, 92.3%, and 84.3%, respectively.

### 5.5. Comparison of Average Departure Time

The average time of departure means that 120 calls are received to the medical staff, and the ambulance is dispatched. The average delivery time of the control group and the experimental group was 1.71 ± 1.62 min and 1.24 ± 1.47 min, respectively. The results of two independent samples *t*-test showed that the prehospital response time of the two groups was compared after the integrated trauma first aid procedure. There was academic significance (*t* = 3.571, *P* ≤ 0.01).

### 5.6. Comparison of Average Arrival Time

The average arrival time is the time during which the ambulance is dispatched to the scene where the injury occurred. The average delivery time of the control group and the experimental group was 8.64 ± 1.31 min and 7.17 ± 1.62 min, respectively. The results of two independent samples *t*-test showed that after the integrated trauma emergency procedure, the average arrival time of the two groups of patients was compared. There was academic significance (*t* = −2.564, *P* = 0.003 < 0.05).

### 5.7. Comparison of Average Transit Time

The mean transit time of the control group and the experimental group was 9.35 ± 1.57 min and 6.53 ± 1.22 min, respectively. The results of two independent samples *t*-test showed that the average transit time of the two groups was compared after the integrated trauma first aid procedure. The difference was statistically significant (*t* = 1.969, *P* = 0.017 < 0.05).

### 5.8. Comparison of Standby Time on Average

The average enrolment time in the control group and the experimental group was 8.37 ± 1.23 min and 6.46 ± 1.29 min, respectively. The results of two independent samples *t*-test showed that after the integrated trauma first aid procedure, the average waiting time of the two groups was compared. There was academic significance (*t* = 2.371, *P* = 0.001 < 0.05).

### 5.9. Comparison of Average Admission to Diversion Time

The time from admission to diversion refers to the time from the admission of the patient to the treatment of emergency treatment, auxiliary examination, hospitalization, and emergency surgery. After the integrated trauma first aid procedure, the difference between the two groups of patients admitted to the shunt time was statistically significant (*H* = 10.729, *P* = −0.001 < 0.05) (Table 3).

### 5.10. Comparison of Treatment Outcomes between the Two Groups of Patients

Using the integrated trauma first aid procedure, the difference in the efficacy of the two groups of patients was statistically significant (*H* = 10.667, *P* = 0.001 < 0.05), as shown in Table 4.

### 5.11. Comparison of Family Satisfaction Scores between the Two Groups

The total score of satisfaction of family members for the application of the integrated trauma first aid procedure was 7.93 ± 0.59 points, while the total score of the traditional first aid satisfaction was 5.87 ± 0.43 points; the difference was statistically significant (*P* < 0.05) (Table 5).

## 6. Conclusion

Based on the process reengineering theory, under the WSN measurement and medical information system, the methods of system reintegration and partial process reengineering are comprehensively used to establish the complete process of the trauma first aid procedure. The results show that WSN measurement and medical information system process reengineering can optimize the treatment process of emergency patients, resulting in significant differences in curative effects (*P* < 0.05). Besides, DBN in deep learning was applied to predict the optimal route of emergency ambulances in the process of first aid, which could realize the prediction of a traffic network. It could be effectively applied in the first aid of emergency patients, which could shorten the time before the triage of emergency patients and improve the satisfaction of patients and their family members.

However, some deficiencies still remain, such as the relatively limited measurement indicators selected. Therefore, further research should be carried out, and evaluation indicators should be added to make a more comprehensive evaluation of the application effect of the integrated trauma first aid process, to improve the quality of emergency medical treatment. Moreover, the first aid system is only used in the surgical first aid process. For the patients who are admitted to the emergency department and go through the hospitalization procedures, they will not be able to continue to be included in the system for redistribution. It will be that the issue needs to be improved in the hospital information management system, so that the patient information in the hospital can be integrated as much as possible.

## Figures and Tables

**Figure 1:** Roadmap for building an integrated trauma emergency process.

**Figure 2:** Traditional trauma first aid flowchart.

**Figure 3:** New process.

**Figure 4:** The basic structures of the restricted Boltzmann machine and the DBN model.

**Figure 5:** First aid route optimization process.

**Figure 6:** Prediction results of the emergency route based on deep learning: (a) accuracy of *T*_0_; (b) accuracy of *W*_*i*_; (c) accuracy of *V*_*i*_.

**Table 1:** Comparison of general conditions and injuries between the two groups of patients (*n* (%)).

Variable	Category	Control group (*n* = 131)	Test group (*n* = 127)	*χ* ^2^	*P*
Gender	Male	91 (69.47)	93 (73.23)	0.274	0.605
	Female	40 (30.53)	34 (26.77)		
Cause of injury	Car accident	94 (71.76)	91 (72.95)	0.613	0.716
	Fall injury	23 (17.56)	19 (71.65)		
	Other injuries	14 (10.69)	17 (13.39)		

**Table 2:** Comparison of wound index scores between the two groups (*n* (%)).

Score	Control group (*n* = 131)	Test group (*n* = 127)	*χ* ^2^	*P*
2~9	79 (60.31)	77 (60.63)	0.469	0.931
10~17	32 (24.43)	33 (25.98)		
17~20	12 (9.16)	12 (9.45)		
20 or more points	8 (6.11)	5 (3.94)		

**Table 3:** Comparison of two groups of patients admitted to the shunt time (*n* (%)).

Group	Within 10 min	Within 20 minutes	Within 30 minutes
Experimental group (*n* = 127)	83 (65.35)	38 (29.92)	6 (4.72)
Control group (*n* = 131)	56 (42.75)	65 (49.62)	10 (7.63)
*H*	10.729		
*P*	0.001		

**Table 4:** Comparison of treatment effects between the two groups of patients (*n* (%)).

Group	Get well	Better	Invalid
Experimental group (*n* = 127)	71 (55.91)	42 (33.07)	14 (11.02)
Control group (*n* = 131)	44 (33.59)	71 (54.20)	16 (12.21)
*H*	10.667		
*P*	0.001		

**Table 5:** Comparison of family satisfaction scores between the two groups of patients (*n* ± *x*).

Group	Medical work attitude	First aid program	Treatment effect	Overall score
Experimental group (*n* = 127)	2.71 ± 0.53	3.01 ± 0.27	3.65 ± 0.35	7.93 ± 0.59
Control group (*n* = 131)	0.23 ± 0.16	2.11 ± 0.54	2.52 ± 0.51	5.87 ± 0.43
*t*	5.217	3.264	2.247	2.551
*P*	≤0.01	≤0.01	0.001	0.001

## Data Availability

The data used to support the findings of this study are available from the corresponding author upon request.
